# How Do Housing Prices Affect Residents' Health? New Evidence From China

**DOI:** 10.3389/fpubh.2021.816372

**Published:** 2022-01-13

**Authors:** Hui-Qin Wang, Li-Qiu Liang

**Affiliations:** College of Economics and Management, Nanning Normal University, Nanning, China

**Keywords:** housing prices, mental health, physical health, promoting effects, inhibitory effects

## Abstract

This paper aims to explore the effect and mechanism of rising housing prices on residents' physical and mental health. Using data from the China Family Panel Studies from 2014 to 2018, we investigate the impact and mechanism of rising housing prices on the mental and physical health of urban residents through multiple grouping regression and analysis of variance. The study finds that overall, rising housing prices have a positive effect on residents' mental health but a negative effect on physical health, and those who do not own a house show the greatest adverse effect. The impact of rising housing prices on health is mainly reflected in three aspects: the wealth effect, cost effect, and comprehensive environmental expectation effect. Of these, the wealth effect and comprehensive environmental expectation effect play a role in promoting residents' health, whereas the cost effect has a strong inhibitory effect. This paper also analyzes how house prices impact health and finds that having health insurance reduces residents' active health behavior, thus affecting their physical and mental health levels, which has a positive effect on uninsured residents.

## Introduction

This paper aims to explore the effect and mechanism of rising housing prices on residents' physical and mental health. Housing is closely related to city residents' sense of belonging, sense of security, children's school attendance, and registered residence in China. Since the reform of China's housing system in 1998, the real estate industry has developed rapidly. The average selling price of commercial housing in China rose from 4,725 yuan/m^2^ in 2010 to 9,980 yuan/m^2^ in 2020 as Figure 1 shows. Housing has become an important asset of urban households with rising prices. According to the 2020 China Household Finance Survey^1^ report, China's urban household housing ownership rate has reached 89.68%, far higher than the market imagination and the world average. At the same time, high housing prices have formed a heavy burden to ordinary residents, not only reflected in their economic level but also impacting their mental and physical health.

**Figure 1:** Change trend of housing price and housing price growth rate (2010–2020). Data source: China's National Bureau of Statistics.

So how do housing prices affect residents' physical and mental health? From the perspective of reality and theory, a close internal relationship exists between housing prices and urban residents' health. First, for residents who already own houses and have no mortgage (or have a strong ability to repay loans), rising housing prices increase the per capita wealth of families, producing the wealth effect of physical and mental health. Second, for residents with housing difficulties, a high proportion of income allocated to paying a mortgage, and low income levels, buying just-needed real estate leads to a substantial increase in the cost of living. The resulting cost effect reduces residents' disposable income and investment in health management, thus damaging their physical and mental health. Finally, the higher the housing prices, the better a city's economic development; infrastructure; and education, medical, and other comprehensive environment. The expected effect of the comprehensive environment has a significant impact on residents' physical and mental health.

Based on this, this paper uses data from the China Family Panel Studies (CFPS) in 2014, 2016, and 2018, combined with China's economic and cultural institutional environment through multiple group regression comparison and analysis of variance. It investigates whether rising housing prices influence residents to change their living conditions and affect their physical and mental health through the wealth effect, cost effect, and comprehensive environmental expectation effect, to provide a theoretical basis for the Chinese government's macro-control and housing price control.

## Literature Review

Many studies focus on how macroeconomic indicators such as economic development and income have an important impact on residents' health levels. Studies find a mutual influence mechanism between income and health, and the amount of income affects the degree of access to resources needed to maintain health (1, 2). D'hombres et al. investigated the income gap impact on health (3), and Acemoglu et al. investigated the effect of government public health investment policy on residents' income (4). Many studies also exist on how housing price fluctuations affect different areas in the economy and society. For example, house prices have a squeezing effect on residents' consumption (5, 6), and high house prices affect population flow (7–9) and female fertility (10, 11), as well as hindering employment, labor mobility supply (12–14), and the entrepreneurial activities of urban adults (15). Aging has an inhibitory effect on house prices (16, 17), the social crime rate increases with the rise of house prices (18), and public service facilities have a direct impact on house prices (19, 20).

The impact of housing price fluctuations on families is mainly from two directions: economic behavior and residents' health. First, housing price fluctuations impact family economic behavior, including consumption and savings. Chen et al. examined the influence of housing price in addition to wealth on consumption in mainland China and believe that real estate price has a significant long-term influence on consumption (21). Chen et al. believe that homeowners who jointly own houses have the highest average consumption tendency, whereas those who independently own houses have the greatest response to the appreciation of housing wealth (22). However, Browning et al. find little evidence of a housing price wealth effect on consumption (23). With insufficient confidence in the future, consumption translates into saving. Chamon argues that savings rates are rising for all population groups because of the increasing burden of private expenditures such as housing, resulting in precautionary incentives that may be amplified by financial underdevelopment, including restrictions on borrowing against future income and low returns on financial assets (24). After controlling for life cycle and other related factors, Wan believes that the growth of housing prices and mortgage loans has a significant positive impact on household savings (25). The second factor is employment. Fu believes that the change of housing value has a significant impact on the probability of female homeowners joining the labor force but little impact on male labor force participation (26). Rabe et al. find that the difference in housing price levels is an important determinant of British household migration where the householder's partner is a bound immigrant (27).

Additionally, rising housing prices impact residents' physical and mental health. Ratcliffe documents a positive correlation between house prices and the mental health of homeowners and non-homeowners (28). Using longitudinal data to assess the impact of housing payment problems on the health of homeowners and renters in 27 European countries, Clair finds that housing payment problems are an important risk factor for renters' self-reported worsening health (29). Kadir et al. find that the rise of local housing prices in Australia have a positive impact on the physical health of property owners and a negative impact on the physical and mental health of tenants, and the former could be partly attributed to health-related investments and behaviors (30). Using the huge external changes of housing wealth to study the influence of wealth gain and loss on personal health, Fichera et al. find that higher house prices lead to greater wealth for homeowners, reduce the possibility of several non-chronic health conditions, and improve self-assessed health but have no effect on mental health (31). For homeowners, the increase of wealth affects labor supply and leisure choices, showing that rising house prices enable individuals to reduce work intensity, with corresponding health benefits. In the United States, Yilmazer and Babiarz find that with the reduction of housing wealth relative to total wealth, mental health deteriorates more seriously, psychological stress increases, and the incidence of depression is higher (32). Wei reveals the possible negative consequences of rising house prices on Chinese residents' mental health, which requires the government to make corresponding policies (33).

Among other relevant studies, Zhang believes that house price appreciation has a more significant impact on low-income families and families in the eastern region of China, but housing debt does not affect the role of housing value in subjective well-being (34, 35). Foote finds that the decline of house prices reduces the immigration of homeowners with low net worth, but it has no impact on homeowners with the highest leverage (36).

Most of the existing literature focuses on housing prices and family economic behavior and residents' income and health. Although some studies exist about the impact of housing price fluctuations on residents' health, most focus on the impact of housing wealth appreciation on residents' health and mortgage pressure or of renting on residents' health and other single factors. Additionally, most related existing research is concentrated in developed countries. However, China's real estate market is very different from European and American countries in housing price growth, people's preference for real estate investment, and government control. The impact of housing price fluctuations on the physical and mental health of Chinese residents, the impact mechanism, and the impact angle may be more complex and diverse than in other countries. Presently, little research exists on how housing prices affect the health of urban residents in China, and only a few of the latest studies have begun preliminary exploration. Therefore, based on data from the CFPS from 2014 to 2018, combined with China's economic and cultural institutional environment through multiple group regression comparison and analysis of variance, we investigate the complex impact of urban housing prices on residents' physical and mental health and test the mechanism.

## Theoretical Analysis and Assumption

Theoretically and practically, housing prices may affect residents' health through the three channels: a wealth effect, cost effect, and comprehensive environmental expectation effect.

### Wealth Effect

As an asset of property owners, rising housing prices bring increased property value, and homeowners experience physical and mental benefits due to the increased total real estate and family net assets. This is reflected in several effects. First, the wealth of homeowners increases, their budgetary expenditure constraints are relaxed, and their investment in health management can be increased to improve their physical and mental health (28). Second, the wealth obtained from the realization or mortgage of real estate increases family assets and turns them into leisure and relaxation consumption expenditure, which plays a positive role in promoting physical and mental health. Third, for residents who own houses and do not need to pay a mortgage, work pressure is relatively low, so they can shorten their working hours and increase their investment in health management to improve their mood and reduce the occurrence of disease (32). Therefore, this paper puts forward the following assumptions:

H1: Rising housing prices have a positive wealth effect on the mental health of urban residents with houses.
H2: Rising housing prices have a positive wealth effect on the physical health of urban residents with houses.

### Cost Effect

Rising house prices increase not only the cost of purchasing basic housing in the future but also the cost of renting and the psychological pressure of residents living in other people's homes, which affects their quality of life. This is reflected in several effects. First, the rise in housing prices leads to demand that cannot be met for improved quality of life for the homeless in areas with little housing, bringing psychological anxiety. Second, increased housing costs directly affect the living consumption level of residents, reduce their investment in health management, and increase their risk of disease. Third, to increase family savings and buy a house as soon as possible, residents extend their working hours or increase their work intensity to obtain higher income and work benefits. This includes the prevalence of “internal roll”^2^ and “996” and “007” working systems,^3^ which are harmful to health (37). Based on this, the following assumptions are made:

H3: Rising house prices have a negative cost effect on the mental health of urban residents without housing.
H4: Rising house prices have a negative cost effect on the health of urban residents without housing.

### Comprehensive Expected Effects of Environment

Housing prices are an important reflection of a region's economic development level and urban vitality. Areas with high housing prices often provide residents with better living conditions, with a significant impact on their physical and mental health. This is reflected in two effects. First, cities with higher housing prices have higher quality social environments, such as better infrastructure, medical conditions, and educational resources, which can have a positive effect on residents' physical and mental health (38). Second, housing prices reflect residents' confidence in their expectations and future. Rising housing prices mean that the region has better development prospects and residents have more space to improve their wealth, thus improving their mental health and increasing their investment in health management (39). Therefore, this paper puts forward the following assumptions:

H5: Rising house prices have a significantly promoting comprehensive environmental expected effect on the mental health of urban residents.
H6: Rising house prices have a significantly promoting comprehensive environmental expected effect on the health of urban residents.

Based on the above theoretical analysis and assumptions, we construct the theoretical model as Figure 2.

**Figure 2:** Theoretical model construction.

## Measurement Models, Data Sources, and Variable Definitions

### Econometric Model Setting


(1) $$\begin{array}{r} Y_{cit}\;=\;\alpha +\beta lnhp_{c,t-1}+\gamma X+u_{cit} \end{array}$$

This paper mainly studies the impact and mechanism of housing prices on residents' health and adopts econometric regression models such as model (1) in empirical analysis. Within these, α, β, and γ are parameters to be estimated and represent random perturbation terms. In the formula, the explained variables Y_cit_ are the physical and mental health status of i residents in province c in the year t under investigation, represented by housing price as the logarithm of the average selling price of residential commercial houses in province c where resident i resides in the year (t−1),^4^ represented by lnhp_c,t−1_. We also control three kinds of variables: personal characteristics, personal family characteristics, and personal province characteristics, expressed by vector X. To accurately estimate the effect, endogeneity problems such as omitted variables and reverse causality should be considered when setting the model. We need to find an appropriate instrumental variable. This variable is the exogenous source of housing price changes and affects the physical and mental health of urban residents through and only through housing prices. Therefore, the two-stage least square method is used to generate instrumental variables to test the endogeneity problem.


(2) $$\begin{array}{r} lnhp_{c,t-1}\;=\;\alpha +\beta w_{ci} \end{array}$$

(3) $$\begin{array}{r} \hat{\;lnhp_{c,t-1}}\;=\;\alpha +\beta w_{ci} \end{array}$$

(4) $$\begin{array}{r} Y_{cit}\;=\;\alpha +\beta lnhp_{c,t-1}+\left[\beta \left(lnhp_{c,t-1}\hat{-lnhp_{c,t-1}}\right)\right]\\ +\gamma X+u_{cit}lnhp_{c,t-1} \end{array}$$

(5) $$\begin{array}{r} F\left(n\right)\;=\;\frac{SST}{SSE} \end{array}$$

Hypothesis: in the first stage, model 2 is constructed through the parameters estimated by Ordinary Least Square, where w is the instrumental variable, and α and β are the demand parameters. In the second stage, α and β are estimated through model 2, then model 3 is fitted. Model 1 is converted into model 4, and OLS is used again to test whether instrumental variables are correlated with explanatory variables.

When analyzing the three effects of housing price on residents' physical and mental health, a comprehensive environmental expected effect test involving a variable of a variety of levels of observation, the influence of the univariate analysis of variance is adopted. The *F* test concludes that housing prices and the comprehensive environmental expected effect of multiple variables impact the health of residents at the same time.

As in model 5, SST is the sum of squares of total effects, and SSE is the sum of squares of deviations between groups. The larger the *F* value, the smaller the influence of the multi-factor variables on observed variables, and vice versa. The associated SIG value is less than the significance level, and the influence is more significant.

### Data Sources and Variable Definitions

The micro data used in this paper are from the CFPS implemented by the China Social Science Survey Center of Peking University in 2014, 2016, and 2018. The research object is limited to the sample of urban residents over 16 years old, and samples with missing values such as personal characteristics are excluded. The total number of mixed section samples in phase III is 51,258. The key variable housing price data come from the China Statistical Yearbook in 2014 and 2018, and the interpreted variable is residents' health status, including self-rated physical and mental health status. Psychological health is measured by the simple average of CES-D, and the higher the value, the better the health status. Because the CFPS data adopts the rotation survey method, the same psychological scale problems exist for 2016 and 2018. The mental health analysis extracts the common parts of the 2014 scale items and the CES-D scale items in 2016 and 2018. The scale includes items such as “I feel depressed,” “I feel it is difficult to do anything,” “My sleep is not good,” “I feel that life is meaningless” (reverse), and “I feel that daily life cannot continue.” The respondents choose the grade according to the description: 1 (almost none), 2 (rarely sometimes), 3 (sometimes), 4 (often), and 5 (mostly). The five physical health questions are used as measuring variables: “self-assessment of physical health status,” “recent changes in health status,” “recent physical discomfort,” “degree of physical illness and injury,” and “chronic disease.” First, for the question “How do you think your health status is?”, the five options are “unhealthy,” “average,” “relatively healthy,” “healthy,” and “very healthy,” with values ranging from 1 to 5. The change in health status is measured on a scale of 1–3, meaning “worse,” “no change,” and “better.” The degree of disease and injury is assigned 0–3 in order from “no disease and injury” to “serious,” and the remaining two variables are binary. If the answer is “yes,” the value is assigned 1, and if the answer is otherwise, it is assigned 0. SPSS26.0 and Stata15.1 software are used to process the data.

Other control variables affecting residents' health status include their personal, family, and regional characteristics. Demographic characteristics include sex and age (1 = male; 0 = female), marriage (1 = married; 0 = unmarried), education (1 = illiterate; 2 = elementary school; 3 = high school; 4 = college degree; 5 = master's or doctoral degree), employment status (1 = employed; 0 = no job), health insurance (1 = have; 0 = none), housing subsidy (1 = yes; 0 = none), medical treatment behavior (1 = yes; 0 = none), late sleep (1 = yes; 0 = no), and weekly exercise duration. Household characteristics include home ownership (1 = owning; 0 = none), housing loan (1 = yes; 0 = none), housing area size (1 = small apartment; 2 = medium; 3 = large house type), total family property, and family net assets. We eliminate the samples lacking property right types and with “other” types; defined family members with full property rights, partial property rights as owning houses; and defined low-rent housing, public housing, commercial housing, and the houses of relatives and friends as not owning houses (rented houses). Regional characteristics include future confidence (1 = very low confidence; 2 = low confidence; 3 = average; 4 = confident; 5 = very confident), urban level (1 = low; 2 = medium; 3 = high),^5^ per capita disposable income, and number of urban health technicians per 10,000 people. All of the descriptive statistics variables are shown in Table 1.

**Table 1:** Descriptive statistics.

**Variables**		**Total sample**				
		**Total**	**Min**	**Max**	**Mean**	**Std.Dev**
	Housing price	51,258	3,629	34,117	7,681.10	5,328.56
	Per capita land transfer area	51,258	0.36	8.23	1.72	0.94
The physical and mental health	Assess mental health (CES-D)	51,258	5	48	10.6	5.02
	Self-assessment of physical health status	51,258	1	5	2.74	1.25
	Recent changes in health status	51,258	1	3	1.79	0.61
	Recent physical discomfort	51,258	0	1	0.29	0.45
	Degree of physical disease and injury	51,258	0	3	0.62	1.03
	Prevalence of Chronic diseases	51,258	0	1	0.21	0.41
Personal characteristics	Age	51,258	16	102	46.44	16.25
	Gender	51,258	0	1	0.48	0.50
	Marriage	51,258	0	1	0.82	0.39
	The degree of education	51,258	1	5	2.43	1.09
	Employment	51,258	0	1	0.66	0.47
	Health care	51,258	0	1	0.93	0.26
	Housing subsidies	51,258	0	1	0.02	0.14
	Medical treatment behavior	51,258	0	1	0.21	0.41
	Stay up late	51,258	0	1	0.34	0.47
	Length of exercise per week	51,258	0	105	3.62	7.03
Family characteristics	Housing ownership	51,258	0	1	0.88	0.33
	Housing loan	51,258	0	1	0.12	0.32
	Number of real estate	51,258	0	8	1.17	0.71
	Housing area	51,258	1	3	2.34	0.80
	Total family estate	51,258	0	8	1.17	0.71
	Household net worth	51,258	0	50,000,000	715,847.69	1,451,563.48
Regional characteristics	Future confidence	51,258	1	5	4.01	0.98
	City level	51,258	1	3	2.36	0.76
	Per capita disposable income	51,258	19,873	62,596	31,378.61	9,721.05
	Number of health technicians available	51,258	48	220	102.27	19.65

The omission of variables can lead to endogeneity problems, and this paper may omit some non-observable variables that change over time, which are related to both housing prices and residents' health but are difficult to measure. Therefore, we need to find an appropriate tool variable. This paper holds that the per capita land transfer area^6^ of the last year is a suitable instrumental variable of housing prices. In the robustness test, this paper further alleviates this problem by eliminating floating population samples and age samples with less influence.

## Analysis of Empirical Results

### Influence of Housing Prices on Physical and Mental Health of Urban Residents

Table 2 shows the OLS regression results of instrumental variables of the impact of housing prices on the physical and mental health of urban residents in China.^7^ After controlling the endogenous bias, housing prices have a significant promoting effect on urban residents' mental health and an inhibiting effect on the whole sample average physical health after controlling the basic individual characteristic variables. First, in theory, rising housing prices have a negative impact on the physical and mental health of residents without housing. The results in column 4 in the table are generally consistent with this theory. For residents without housing and mortgages, the rise of housing prices has no significant impact, but for each 10% increase inhousing prices, the probability of residents reporting illness increases by 6.5%. Second, for residents with houses and mortgages, rising housing prices have a positive impact on their psychological state, but the effects of various physical health measurement variables are not consistent. As shown in column 2 of the table, rising housing prices have no significant correlation with residents' recent physical changes and chronic diseases but have a significant negative impact on self-rated physical health status. Third, for residents who have houses without mortgages, rising housing prices have a positive effect on their physical and mental health.

**Table 2:** The influence of housing price on physical and mental health of urban residents.

**Variables**	**(1)**	**(2)**	**(3)**	**(4)**	**(5)**
	**All the samples**	**Own houses**		**Without houses**	
		**With mortgage**	**Without mortgage**	**With mortgage**	**Without mortgage**
Assess mental health	0.017 (17.277)^***^	−0.103 (7.979)^***^	0.072 (14.37)^**^	−0.091 (−1.142)	0.024 (1.711)^*^
Self-assessment of physical health status	−0.027 (−6.278)^***^	−0.038 (−2.896)^**^	0.026 (−5.252)^***^	−1.10 (1.951)^*^	−0.005 (−0.411)
Recent changes in health status	−0.05 (−1.146)	0.019 (1.457)	−0.009 (−1.84)^*^	1.41 (−2.483)^**^	0.023 (1.783)^*^
Recent physical discomfort	−0.031 (−7.129)^***^	−0.046 (−3.445)^***^	−0.025 (−4.941)^***^	−1.71 (−3.018)^***^	−0.065 (−5.084)^***^
Degree of physical disease and injury	−0.34 (−7.735)^***^	−0.042 (−3.162)	−0.028 (−5.599)^***^	−1.5 (−2.648)^***^	−0.07 (−5.535)
Prevalence of chronic diseases	−0.03 (−0.653)	0.006 (0.456)	−0.001 (−0.212)	−0.025 (0.425)	−0.025 (−2.022)^***^

*The brackets in the table are T test values*,

*, ** and *** *indicate excessive at the level of 10, 5, and 1% respectively. “Without houses but with mortgage” refers to residents who have no property ownership record under their name, but have a previous loan record (stop offering the house for sale) or who have no registered property ownership but take out a loan in their own name*.

Overall, we find that rising housing prices have a positive effect on the mental health of Chinese urban residents but an inhibitory effect on physical health. In the subsample, the adverse effect on mental health is possibly due to the economic stress caused by mortgage repayment, which increases the risk of mental illness among residents without mortgage stress. The positive impact on physical health is possibly because rising housing prices can promote the improvement of residents'consumption level, increase investment in health management, and improve the living environment.

### Analysis of the Impact of Housing Prices on Urban Residents' Health

How do medical care and health behaviors work to improve health? We continue our analysis to further explain the impact of housing prices on residents' health.

We divide our sample into those with and without health insurance. The corresponding regression results are reported in Table 3. VIF test values of all results are close to 1, with no multicollinearity of the measured variables. These results indicate that regardless of whether residents have insurance, increased housing prices have an inhibitory effect on their medical treatment behavior, but this is insignificant for those without insurance.

**Table 3:** The way analysis of the impact of housing price on urban residents' health.

**Variables**		**Have health insurance**	**No health insurance**
Medical treatment behavior	LN (House prices)	−0.035 (−7.714)^***^	−0.018 (1.147)
Stay up late	LN (House prices)	0.089 (20.109)^***^	0.078 (4.959)^***^
Length of exercise per week	LN (House prices)	−0.02 (−4.49)^**^	0.016 (0.949)

*The brackets in the table are T test values*,

** and *** *indicated excessive at the level of 5, and 1% respectively*.

The regression results for health behavior show that with increased housing prices, residents have an increased probability of sleeping late due to anxiety and other negative emotions, which affect health behavior. For those with health insurance, a 10% increase in housing prices is associated with an 8.9% increase in the likelihood of staying up late and a 2% decrease in the amount of time spent exercising. Staying up late for a long time harms mental state and stability and interferes with initiating normal healthy behaviors, thus endangering the health of urban residents, and the adverse impact on uninsured residents is more significant. Residents with health insurance, which already shares most of the cost of medical care, can bear the negative pressure of rising housing prices and are more likely to relax their health management and neglect physical exercise. However, residents without insurance must bear all expenses if they fall ill, which is a heavy burden. They pay more attention to physical exercise and improving their fitness to reduce the chance of seeking care when they fall ill. Therefore, it has a positive effect on active exercise.

In general, health insurance has a negative effect on residents' physical and mental health through health behaviors, especially for residents who have no kind of health insurance.

### Examining the Effect Mechanism of Housing Priceson Urban Residents' Health

#### Wealth Effect

Does a wealth effect exist for homeowners? In this paper, the samples with houses are divided into those with and without mortgages. Comparative analysis is conducted according to the number of houses, total household properties, and net assets of families to test whether a wealth effect exists. The results are shown in Table 4.

**Table 4:** The wealth effect of housing price on residents' physical and mental health.

**Variables**	**With mortgage**			**Without mortgage**		
	**Number of real estate**	**Total family estate**	**Household net worth**	**Number of real estate**	**Total family estate**	**Household net worth**
Assess mental health	0.025 (4.571)^***^	−0.059 (−5.351)^***^	0.056 (−5.176)^***^	−0.053 (−4.070)^***^	1.17 (−3.410)^**^	0.029 (0.856)
Self-assessment of physical health status	0.003 (0.575)	−0.027 (−2.544)^**^	0.01 (0.968)	0.009 (0.65)	−0.007 (−0.1998)	0.003 (0.086)
Recent changes in health status	0.01 (2.02)^**^	0.003 (0.319)	−0.004 (−0.374)	0.027 (1.865)^***^	0.001 (0.026)	0.001 (0.038)
Recent physical discomfort	−0.002 (0.341)	−0.009 (−0.866)	−0.019 (−1.743)	−0.2 (−1.342)	0.005 (0.123)	−0.009 (−0.241)
Degree of physical disease and injury	−0.003 (−0.565)	−0.022 (−2.056)	0.012 (−1.094)	−0.02 (−1.372)	0.005 (0.13)	−0.058 (−1.636)
Prevalence of chronic diseases	−0.01 (−2.093)^***^	0.011 (1.033)	−0.002 (−0.236)	0.024 (1.667)^*^	−0.022 (−0.627)	0.026 (0.737)

*The brackets in the table are T test values*,

*, ** and *** *indicated excessive at the level of 10, 5, and 1% respectively*.

For residents with houses and mortgages, the number of houses has a negative impact on mental health. With increasing housing prices, the amount and value of real estate increase in proportion, but the mortgage burden also increases, increasing the risk of mental illness. Among the five variables measuring physical health, only the number of houses has a significant positive effect on residents' self-rated health (*p* = 0.058). With an increase in housing price of 10%, the probability that residents think their health condition will get better increases by 2.7%, whereas some residents think it will increase the risk of chronic diseases, which has adverse effects.

For residents who own houses but do not have mortgages, the number of houses has a strong positive effect on mental health and a significant positive effect on the perception of physical health and the incidence of chronic diseases. Real estate value and family net worth have significant inhibitory effects on residents' mental health. This is because increased housing prices have a wealth effect on rising property values and household assets. However, China's market has many constraints on the flow and change of real estate. Regulation policies, such as restrictions on sales and loan suspensions of second-hand houses, make residents who want to use their surplus real estate for investment or cash face the risk of loss, so they are more prone to worry, anxiety, and other negative emotions. The influence of property value on physical health is inconsistent. The more total property, the lower the health level, due to physical problems caused by psychological factors. However, an increased value of assets and real estate correspondingly improves the living standards of residents, and the degree of illness and injury is also improved.

In general, as housing prices rise, the number of houses has a wealth effect on physical health, which is in line with hypothesis H2. For residents with houses and mortgages, the number of houses also has a wealth effect on their mental health, which is partially consistent with hypothesis H1, but the effect on physical health is offset by a negative cost effect. Therefore, rising housing prices do have a wealth effect on the health of urban residents with houses, but this does not play a leading role.

#### Cost Effect

Will the continuous rise in house prices have a negative cost effect on those without homes? The results of the inspection and analysis are shown in Table 5. Rising housing prices have a significant adverse effect on the mental health of residents who do not own houses or have mortgages. The smaller the housing area, the worse the living standard and health condition. For residents with mortgage pressure, their physical discomfort (*p* = 0.034) and degree of illness and injury (*p* = 0.037) significantly increased, but the housing subsidy can compensate the burden of housing expenses. In general, when housing prices rise, this has a significant cost effect on the health of urban residents without houses, which conforms to hypotheses H3 and H4. The adverse impact on mental health is the greatest for residents with mortgage pressure.

**Table 5:** The cost effect of housing price on residents' physical and mental health.

**Variables**	**Housing area**	**Mortgage**	**Housing subsidies**
Assess mental health	−0.09 (−1.5)	−0.062 (−4.959)^***^	−0.001 (−0.043)
Self-assessment of physical health status	0.035 (2.825)^***^	0.356 (0.92)	0.02 (1.615)
Recent changes in health status	0.029 (2.353)	0.002 (0.123)	−0.009 (0.368)
Recent physical discomfort	−0.046 (−3.63)^***^	0.026 (−2.123)^**^	−0.009 (0.688)
Degree of physical disease and injury	−0.039 (−3.101)^***^	0.058 (−2.083)^**^	−0.006 (−0.518)
Prevalence of chronic diseases	−0.021 (−1.758)	0 (−0.031)	−0.117 (−5.533)

*The brackets in the table are T test values*,

** and *** *indicated excessive at the level of 5, and 1% respectively*.

#### Comprehensive Expected Effects of Environment

Housing price levels reflect the economic vitality of a region, the level of development, and other comprehensive environment signals. If the expected effect of comprehensive environment does exist, housing prices will have different degrees of impact on residents. Because multiple variables are involved to test the health measurement variables, one-way analysis of variance is adopted in this paper, and the results are shown in Table 6.

**Table 6:** Comprehensive expected effect of housing price on residents' physical and mental health.

**Variables**	**(1)**	**(2)**	**(3)**	**(4)**	**(5)**	**(6)**	**(7)**	**(8)**
	**Future confidence**		**City level**		**Per income**		**Health technicians**	
	**M**	**I**	**M**	**I**	**M**	**I**	**M**	**I**
Assess mental health	106.983^***^	3.954^***^	304.768^**^	1.512^**^	361.666	0.041	365.436	0.041
Self-assessment of physical health status	9.393^***^	0.48	7.784^***^	1.377^*^	9.118^***^	0.48^*^	9.207^***^	0.48^*^
Recent changes in health status	6.803^***^	2.442^***^	5.719^***^	0.892	6.695^***^	0.417	6.742^***^	0.417
Recent physical discomfort	5.234^***^	2.653^***^	5.472^***^	1.44	6.270^***^	0.940	6.336^***^	0.940
Degree of physical disease and injury	6.30^***^	2.915^***^	5.657^***^	0.865	6.582^***^	1.234	6.651^***^	1.234
Prevalence of chronic diseases	6.243^***^	2.83^***^	6.691^***^	0.862	7.797^***^	1.043	7.879^***^	1.043

*In this table, Per income on behalf of the per capita disposable income, Health technicians on behalf of the number of health technicians available, M on behalf of the model, I on behalf the Interaction. The brackets in the table are T test values*,

*, ** and *** *indicated excessive at the level of 10, 5, and 1% respectively*.

The F value of the model analysis of variance results is large, and the *p* < 0.05, indicating that the model is effective. From the results of the interactive analysis, a causal relationship exists between the comprehensive environmental expected effect and residents' physical and mental health when house prices rise. The interaction between future confidence and housing prices has a significant impact on residents' physical and mental health. Rising housing prices mean that residents have more confidence in the future development of the city and their own future development, which has a positive implication on the psychological level and promotes physical health. The interaction between the urban comprehensive environment and housing prices has a significant effect on residents' health, especially for the overall health status evaluation. The higher the level of urban development, the larger the corresponding increase of housing price, and the stronger the positive effect of urban public services. Both measurement variables support hypothesis H5 and H6. The interaction between per capita disposable income and housing prices has no significant effect on mental health, although the greater per capita disposable income, the more positive mood reported. However, prolonged working hours, such as “996” and “007” overtime models, can easily cause serious harm to residents' health. In general, when housing prices rise, improved urban public service level and residents' confidence in the future can significantly promote the expected effect of the comprehensive environment, but there are other factors in the comprehensive environment that will damage the physical and mental health of residents, thus partially offset the promotion effect to residents' health.

### Robustness Test

Next, we remove samples from the floating population and of inapplicable age to mitigate selective bias. Principal component analysis is used to alleviate the measurement errors of physical and mental health in the explained variables.

#### Sample Bias Problem

Although this paper partly controls the attraction of cities to the floating population by controlling several personal characteristics, it cannot deal with this problem completely. Due to data limitations, this paper can only eliminate samples of the floating population and unsuitable age (under 20 and over 65 years old) to alleviate the endogeneity problems caused by sample bias. As Table 7 shows, increased housing prices reduce the health level of residents but reduce their physical discomfort and degree of illness and injury, which may be due to the comprehensive environmental expectation effect. The higher the level of regional economic development, the better the medical conditions, which is more conducive to the prevention and cure of diseases.

**Table 7:** Sample bias problem.

**Variables**	**Self-assess of mental health**	**Self-assessment of physical health**				
		**Self-assessment of physical health status**	**Recent changes in health status**	**Recent physical discomfort**	**Degree of physical disease and injury**	**Prevalence of Chronic diseases**
LN (House prices)	−0.085 (−16.028)^***^	−0.026 (−5.055)^***^	−0.003 (−0.566)^***^	−0.036 (−6.615)^***^	−0.036 (−5.058)^***^	−0.006 (−1.057)^***^

*The brackets in the table are T test values*,

*** *indicated excessive at the level of 1%*.

#### Measurement of Physical and Mental Health

Although self-rated health is used as a reflection of individuals' actual health status in many studies, some scholars think this is not objective enough. Therefore, this paper synthesizes five measurement variables of physical health and obtains comprehensive indicators of physical health^8^ through principal component analysis. The same applies to mental health.^9^

The results in Table 8 show the corresponding regression results. Housing price increases significantly improve the physical and mental health of residents with houses and have a negative effect on the physical and mental health of residents without houses. For every 10% increase in housing prices, the mental health level of homeowners increases by 1.5%, whereas that of non-homeowners decreases by 7.8%. The physical fitness of homeowners increases by 5%, whereas that of non-homeowners decreases by 5.4%.

**Table 8:** Principal component physical and mental health measurement.

**Variables**	**Mental health**		**Physical health**	
	**Own houses**	**Without houses**	**Own houses**	**Without houses**
LN (House prices)	0.015 (−12.831)^***^	−0.078 (−6.189)^***^	0.05 (−1.5)^***^	−0.0254 (−4.465)^***^

*The brackets in the table are T test values*,

*** *indicated excessive at the level of 1%*.

## Conclusions and Policy Recommendations

This paper uses the data from the CFPS in 2014, 2016, and 2018 to explore the impact of housing price changes on residents' health status, using an econometric regression model. We find that housing price changes affect residents' lifestyles through a wealth effect, cost effect, and comprehensive environmental expectation effect, there by affecting their physical and mental health. On the whole, rising housing prices promote the mental health of residents but some what inhibit their physical health. Residents without houses show the greatest adverse impact. Having health insurance reduces physical and mental health by affecting the daily health behavior of residents, and the negative impact is more significant for the uninsured. Among the three mechanisms, the wealth effect and the comprehensive environmental expectation effect play a role in promoting health, while the cost effect plays a strong role in inhibiting it. This study confirms the important impact of rising housing prices on residents' health.

Housing and health are two of the greatest concerns for China. In recent years, the real estate market has continued to grow. Although its contribution to household wealth has declined slightly after the COVID-19 pandemic, it is still a key factor. Given the significant impact of China's macro economic regulation on housing prices, the government should remain sensitive to changes in urban housing prices, strengthen the regulation and control of the real estate market, restrain housing prices from rising too quickly, and meet rigid housing demands. Policy implementation measures should be taken according to local conditions.

## Data Availability Statement

The original contributions presented in the study are included in the article/supplementary material, further inquiries can be directed to the corresponding author.

## Author Contributions

H-QW: conceptualization, methodology, and writing and reviewing. L-QL: software and data preparation. All authors contributed to the article and approved the submitted version.

## Funding

This research is partly supported by the National Social Science Fund of China (20BJL087), Philosophy and Social Sciences Fund of Guangxi Province (21CJY013).

## Conflict of Interest

The authors declare that the research was conducted in the absence of any commercial or financial relationships that could be construed as a potential conflict of interest.

## Publisher's Note

All claims expressed in this article are solely those of the authors and do not necessarily represent those of their affiliated organizations, or those of the publisher, the editors and the reviewers. Any product that may be evaluated in this article, or claim that may be made by its manufacturer, is not guaranteed or endorsed by the publisher.

## Footnotes

^1^2020 China Household Finance Survey. https://chfs.swufe.edu.cn/.

^2^Involution: refers to the social phenomenon in which people in the same industry make greater efforts to compete for limited resources, and competitive pressure increases, resulting in decreased individual income and effort ratio. It can be regarded as the “inflation” of effort, and the opposite phenomenon is “lying down”.

^3^996 and007: the product of the expansionary development of the 996 working system, which gains greater marginal benefits by extending working hours. This refers to going to work at 9 am and leaving at 9 pm, 6 days a week. Similarly, 007 refers to going to work at midnight and leaving at midnight, 7 days a week.

^4^Since the CFPS survey mainly focuses on July and August, and some health questions ask about the past 6 months, the house price lagging behind the first period is adopted.

^5^The value is assigned according to the latest national provincial GDP ranking.

^6^The per capita land transfer area data are from the Yearbook of China's land and resources from 2014 to 2018.

^7^Because the software output directly obtains the second stage results, the first stage results are lacking.

^8^The KMO of the principal component analysis of the comprehensive indicators of mental health is 0.639, indicating that the principal component analysis is very suitable for many mental health problems.

^9^The KMO of the principal component analysis of the comprehensive indicators of mental health is 0.788, indicating that multiple mental health problems are very suitable for principal component analysis.
